The article "Overexpression of microRNA-203 Suppresses Proliferation, Invasion, and Migration while Accelerating Apoptosis of CSCC Cell Line SCL-1" was retracted in 2022. Reason: concerns about the data.

# Overexpression of microRNA-203 Suppresses Proliferation, Invasion, and Migration while Accelerating Apoptosis of CSCC Cell Line SCL-1

**DOI:** 10.1016/j.omtn.2020.04.014

**Published:** 2020-05-01

**Authors:** Wenyun Ting, Cheng Feng, Mingzi Zhang, Fei Long, Ming Bai

**Affiliations:** 1 Department of Plastic and Aesthetic Surgery, Peking Union Medical College Hospital, Beijing 100730, P.R. China

**Keywords:** microRNA-203, cutaneous squamous cell carcinoma, Wnt/β-catenin signaling pathway, PRC1, apoptosis, invasion

## Abstract

Cutaneous squamous cell carcinoma (CSCC) is a malignant proliferation of cutaneous epithelium that has been observed to have an alarming rise in incidence. Numerous studies have demonstrated microRNAs (miRNAs or miRs) as important biomarkers in the diagnosis, prognosis, and treatment of CSCC. This study aims to investigate the effects of miR-203 on the behaviors of CSCC cells and possible mechanisms associated with protein regulator of cytokinesis-1 (PRC1) and Wnt/β-catenin signaling pathway. PRC1 was suggested as a target of miR-203 in squamous cell carcinoma cell line 1 (SCL-1) cells by dual-luciferase reporter gene assay. Based on the immunohistochemical staining and qRT-PCR, PRC1 was abundantly expressed while miR-203 was poorly expressed in CSCC tissues. miR-203 mimic or inhibitor was transfected into SCL-1 cells to upregulate or downregulate its expression. Upregulation of miR-203 downregulated PRC1 expression to block the Wnt/β-catenin signaling pathway. By conducting 3-(4,5-dimethylthiazol-2-yl)-2, 5-diphenyltetrazolium bromide (MTT), scratch test, and Transwell and flow cytometric analyses, miR-203 was witnessed to restrain SCL-1 cell proliferation, migration, and invasion while accelerating their apoptosis. The rescue experiments addressed that inhibition of the Wnt/β-catenin signaling pathway conferred the anti-tumor effect of miR-203. These results establish a tumor-suppressive role for miR-203 in CSCC cell line SCL-1. Hence, miR-203 has promising potential as a therapeutic target for CSCC.

## Teaser

The study mainly addressed a tumor-suppressive role of miR-203 in cutaneous squamous cell carcinoma cell line SCL-1 and indicated an antitumor mechanism that was associated with downregulation PRC1 and inhibition of Wnt/β-catenin signaling pathway.

## Introduction

Cutaneous squamous cell carcinoma (CSCC) is a malignancy of the skin characterized by the aberrant proliferation of keratinocytes.^1^ It accounts for more than 20% of all skin cancer-related mortality.^2^ Despite the successful eradication in the majority of cases following surgical excision, there still emerged a high rate of recurrence, metastasis, and death in CSCC patients.^3^ Interestingly, microarray data analysis is widely used to identify candidate genes with the potential to function as diagnostic and prognostic markers for CSCC.^4^ Moreover, a growing number of studies have demonstrated the involvement of differentially expressed microRNAs (miRNAs or miRs) in the molecular pathogenesis of CSCC and have highlighted them as excellent candidate biomarkers for the diagnosis, prognosis, and treatment of CSCC.^5^^,^^6^

miRNAs, existing in multicellular eukaryotes, represent small non-coding RNA molecules that are implicated in the development of cancers, including CSCC.^7^ miRNAs play important roles in the regulation of cancer cell invasion, proliferation, and apoptosis.^8^ Functioning as a significant regulator of tumor progression at different periods, miR-203 has been highlighted as a prognostic marker in CSCC since it shares an association with a good prognosis.^9^ Although miR-203 has been found to suppress the proliferation and angiogenesis-inducing capacity of CSCC cells,^10^ the molecular mechanism associated with its anti-tumor function remains to be investigated. Protein regulator of cytokinesis-1 (PRC1), also known as ASE1, is identified to be a mitotic spindle associated cyclin dependent kinases (CDKs) substrate that is involved in cytokinesis.^11^ PRC1 contributes to tumorigenesis in lung adenocarcinoma via the activation of the Wnt/β-catenin signaling pathway.^12^ The Wnt/β-catenin signaling pathway is one of the typical pathways involved in cell signal transduction, in which the phosphorylation of β-catenin is important for the signaling transduction, influencing tumorigenesis, cell multiplication, and differentiation.^13^ Abnormal upregulation of β-catenin has been detected in CSCC samples*.*^14^ The activation of the Wnt/β-catenin signaling pathway plays a significant role in proliferation, metastasis, and apoptosis of oral squamous cell carcinoma (OSCC) cells, both *in vitro* and *in vivo*.^15^ Moreover, the activation of the Wnt/β-catenin signaling pathway has been reported to induce carcinogenesis and the progression of esophageal squamous cell carcinoma*.*^16^ The present study was conducted to examine the potential role of miR-203 in the growth, migration, invasion, and apoptosis of CSCC cells, and whether miR-203 could interact with PRC1 gene and the Wnt/β-catenin signaling pathway.

## Results

### PRC1 Was Selected and Predicted to Be Regulated by miR-203

Gene expression dataset GEO: GSE66359 was downloaded from gene expression omnibus (GEO) database, from which 348 differentially expressed genes were screened, with 154 upregulated and 194 downregulated genes. EphB2 was found to be one of the downregulated genes related to tumor cell proliferation, migration, and invasion from the GSE66359 dataset. EphB2 has been identified as a therapeutic target in invasive skin cancer and the expression of EphB2 is mediated by RAC1.^17^^,^^18^ RAC1 was not found in the differentially expressed genes. However, PRC1, a direct regulator of RAC1 expression, was found in the differentially expressed genes among the dataset and was regarded as a candidate gene. A previous study found that the abnormal expression of PRC1 may predict recurrence of male prostate cancer, which can be used as a marker of prognosis for this malignancy.^19^ However, its role in CSCC remains unclear, making it crucial to study the role of PRC1 in CSCC. Moreover, PRC1 was differentially expressed with a larger fold change among the top differentially expressed genes (Figure 1A). The relationship between expression of PRC1 gene and the prognosis of CSCC was retrieved from the TCGA database (http://ualcan.path.uab.edu/cgi-bin/ualcan-res.pl), the results of which found that the expression of PRC1 was related to the prognosis of CSCC patients (p < 0.05; Figure 1B). Moreover, the overexpression of PRC1 is an indicator of poor survival rate of breast cancer patients.^20^ The miRNAs that could potentially regulate PRC1 were predicted using *in silico* analyses in order to study the upstream of differentially expressed gene PRC1, and the results from the three databases were displayed on a Venn diagram. As depicted in Tables S1, S2, and S3, the miRSearch and microRNA.org databases failed to give combined values and only the miRDB database provided predicted values. In order to narrow the range of candidate miRNAs, we conducted Venn analyses of all the predicted miRNAs from the miRSearch and microRNA.org databases and the predicted miRNAs with scores higher than 80 from the miRDB database. After taking the intersection, only 1 miRNA, named hsa-miR-203 was found from the three predicted results (Figure 1C).

**Figure 1:** The Potential Significance of miR-203 and PRC1 in CSCC (A) A heatmap of differentially expressed genes in GEO: GSE66359 gene-expression dataset. (B) A survival curve of patients with high and low PRC1 expression in CSCC. (C) Venn analysis of the predicted miRNAs that could regulate PRC1 from three databases (miRSearch, miRNA, and miRDB).

### PRC1 Is a Target Gene of miR-203

According to the results from online bioinformation analysis, a binding site existed between miR-203 and 3′ untranslated region (UTR) of PRC1 (Figure 2A), suggesting that PRC1 was a target gene of miR-203. To verify this binding relationship, we performed dual-luciferase reporter assay using SCL-1 cells. SCL-1 cells were transfected with empty vector, or co-transfected with miR-203 mimic and wild-type (WT)-PRC1/mutant (MUT)-PRC1, or with miR-203 mimic and WT-PRC1/MUT-PRC1 in the presence of miScript target protectors. Compared with the empty vector group, the luciferase activity was reduced by approximately 57% in the miR-203 mimic-WT-PRC1 group (p < 0.05). However, the miR-203 mimic-MUT-PRC1 group presented with no significant difference in luciferase activity (p < 0.05) (Figure 2B). Transfection of custom-designed miScript target protectors against the predicted miR-203 target sites in the PRC1 3′ UTR abrogated the effect of the miR-203 mimic. The results suggested that miR-203 was able to bind to PRC1.

**Figure 2:** PRC1 Was Confirmed as a Target of miR-203 (A) Binding sites between miR-203 and the PRC1 3′ UTR predicted by microRNA.org website. (B) The binding of miR-203 to PRC1 in SCL-1 cells confirmed by dual-luciferase reporter gene assay. ∗p < 0.05 versus the empty vector group.

### High Positive Expression of PRC1 Protein in CSCC Tissues

Immunohistochemistry was used to determine the positive expression of PRC1 protein in CSCC tissues and adjacent normal tissues. As shown in Figure 3, the percentage of PRC1 positive cells was 10.42% ± 0.47% in adjacent normal tissues, 15.17% ± 0.62% in highly differentiated CSCC tissues, 21.81% ± 1.08% in the moderately differentiated CSCC tissues, and 43.85% ± 1.88% in poorly differentiated CSCC tissues. These results indicated that highly, moderately, and poorly differentiated CSCC tissues had a higher PRC1 protein expression compared with adjacent normal tissues (p < 0.05). In addition, the PRC1 protein, which appeared to be brown, was found to be mainly expressed in the cytoplasm of the cells around the necrotic region, as well as in the nucleus.

**Figure 3:** PRC1-Positive Expression Was Increased in CSCC Tissues Versus Adjacent Normal Tissues (A) PRC1-positive expression in CSCC and adjacent normal tissues detected by immunohistochemistry (scale bar, 25 μm). (B) Percentage of PRC1-positive cells in CSCC and adjacent normal tissues. ∗p < 0.05 versus adjacent normal tissues.

### PRC1 Is Upregulated and miR-203 Is Downregulated in CSCC tissues

The expression of miR-203, PRC1, and its known target Snail2 in CSCC tissues and adjacent normal tissues was determined by quantitative reverse transcription polymerase chain reaction (qRT-PCR), as well as *in situ* hybridization of miR-203 expression was conducted. As depicted in Figure 4A, compared with adjacent normal tissues, moderately and poorly differentiated CSCC tissues presented with downregulated miR-203 expression (p < 0.05), among which miR-203 had the lowest expression in the poorly differentiated CSCC tissues (p < 0.05). However, there was no evident difference in miR-203 expression between the highly differentiated CSCC tissues and adjacent normal tissues (p > 0.05). As compared to adjacent normal tissues, moderately and poorly differentiated CSCC tissues had upregulated expression of PRC1 (p < 0.05), among which PRC1 expression was highest in poorly differentiated CSCC tissues (p < 0.05). However, no significant difference was observed in PRC1 expression between the highly differentiated CSCC tissues and adjacent normal tissues (p > 0.05). Meanwhile, no significance was observed in the Snail2 expression among those groups (Figure 4A). Consistent downregulation in miR-203 expression was witnessed in the moderately and poorly differentiated CSCC tissues compared to adjacent normal tissues, with lowest miR-203 expression in the poorly differentiated CSCC tissues (Figure 4B). The aforementioned data suggested that PRC1 expression was highly expressed and miR-203 expression was lowly expressed in CSCC tissues.

**Figure 4:** Poor miR-203 Expression and High PRC1 Expression Were Observed in CSCC Tissues (A) miR-203 expression and PRC1 and Snail2 mRNA expression in CSCC and adjacent normal tissues determined by qRT-PCR. (B) Detection of miR-203 expression by chromogenic *in situ* hybridization (scale bar, 25 μm). ∗p < 0.05 versus adjacent normal tissues.

### Upregulation of miR-203 Blocks the Wnt/β-Catenin Signaling Pathway and Downregulates CSCC Cellular Apoptotic Proteins through Targeting PRC1

Gain- and loss-of-function experiments of miR-203 and PRC1 were conducted using miR-203 mimic, miR-203 inhibitor, oe-PRC1, and sh-PRC1 plasmids, respectively. XAV-939, an inhibitor of the Wnt/β-catenin signaling, was utilized to block the Wnt/β-catenin signaling pathway. qRT-PCR and western blot analysis were conducted to measure expression of miR-203, and mRNA and protein expression of PRC1, the Wnt/β-catenin signaling pathway-related factors including β-catenin, Wnt8b, c-Jun, frizzled-3 (FZD3), cell apoptosis-related factors including p16 and B cell leukemia/lymphoma 2 (Bcl-2), and cell proliferation-related factor c-Myc in SCL-1 cells. The results depicted in Figures 5 and 6 displayed that compared with the blank group, the expression of miR-203 was markedly increased in the miR-203 mimic group, miR-203 mimic + XAV-939 group, and miR-203 mimic + oe-PRC1 group, while miR-203 expression was remarkably reduced in the miR-203 inhibitor group, miR-203 inhibitor + XAV-939 group, and miR-203 inhibitor + sh-PRC1 group (p < 0.05). Compared with the blank group, the mRNA and protein expression of PRC1 was decreased in the miR-203 mimic and miR-203 mimic + XAV-939 groups, whereas PRC1 mRNA and protein expression was elevated in the miR-203 inhibitor and miR-203 inhibitor + XAV-939 groups (p < 0.05), with no significant difference observed in the XAV-939 and negative control (NC) groups (p > 0.05). Compared with the blank group, the mRNA and protein expression of β-catenin, Wnt8b, c-Jun, FZD3, Bcl-2, and c-Myc was elevated in the miR-203 inhibitor and oe-PRC1 groups but lowered in the miR-203 mimic, XAV-939, sh-PRC1, and miR-203 mimic + XAV-939 groups (p < 0.05). No notable difference was observed in those mRNAs and proteins mentioned above between the miR-203 mimic group and the XAV-939 group or among the NC, miR-203 mimic + oe-PRC1, miR-203 inhibitor + sh-PRC1, and miR-203 inhibitor + XAV-939 groups (p > 0.05). The expression of β-catenin, Wnt8b, c-Jun, FZD3, Bcl-2, and c-Myc mRNAs and proteins was reduced in the miR-203 mimic + XAV-939 group while that of those mRNAs and proteins was elevated in the miR-203 mimic + oe-PRC1 group when compared with those in the miR-203 mimic group (p < 0.05). As compared to the miR-203 inhibitor group, the miR-203 inhibitor + XAV-939 group and miR-203 inhibitor + sh-PRC1 group exhibited reductions in the expression of β-catenin, Wnt8b, c-Jun, FZD3, Bcl-2, and c-Myc mRNAs and proteins (p < 0.05). The mRNA and protein expression of p16 was reduced in the miR-203 inhibitor group in comparison to the blank group but increased in the miR-203 mimic, XAV-939, and miR-203 mimic + XAV-939 groups (p < 0.05), with no significant difference observed between the miR-203 mimic group and the XAV-939 group (p > 0.05). Also, no significant difference in the p16 expression was witnessed among the NC, miR-203 mimic + oe-PRC1, miR-203 inhibitor + sh-PRC1, and miR-203 inhibitor + XAV-939 groups (p > 0.05). Compared with the miR-203 mimic group, upregulated p16 mRNA and protein expression was determined in the miR-203 mimic + XAV-939 group, while lower p16 mRNA and protein expression was determined in the miR-203 mimic + oe-PRC1 group (p < 0.05). The miR-203 inhibitor + XAV-939 group and miR-203 inhibitor + sh-PRC1 group had higher p16 mRNA and protein expression relative to the miR-203 inhibitor group (p < 0.05). The above results indicated that miR-203 overexpression resulted in the suppression of Wnt/β-catenin signaling pathway activation and reduced expression of pro-apoptotic proteins by targeting PRC1.

**Figure 5:** miR-203 Downregulated β-catenin, Wnt8b, c-Jun, FZD3, Bcl-2, and c-Myc but Upregulated p16 (A) Expression of miR-203 and PRC1 in cells following various transfection determined by qRT-PCR. (B) Expression of the Wnt/β-catenin signaling pathway-related genes β-catenin, Wnt8b, c-Jun, FZD3 in cells following various transfection determined by qRT-PCR. (C) Expression of apoptosis-related genes p16 and Bcl-2, as well as proliferation-related gene c-Myc in cells following various transfection determined by qRT-PCR. ∗p < 0.05 versus the blank group and the NC group; #p < 0.05 versus the miR-203 mimic group; and &p < 0.05 versus the miR-203 inhibitor group.

**Figure 6:** miR-203 Downregulated β-catenin, Wnt8b, c-Jun, FZD3, Bcl-2, and c-Myc Proteins but Upregulated p16 Protein (A) Western blots of β-catenin, Wnt8b, c-Jun, FZD3, p16, Bcl-2, and c-Myc in cells. (B) Quantitative analysis of band intensities following various transfection. ∗p < 0.05 versus the blank group and the NC group; #p < 0.05 versus the miR-203 mimic group; and &p < 0.05 versus the miR-203 inhibitor group.

### Upregulation of miR-203 Inhibits the Viability of SCL-1 Cells

The cell viability of SCL-1 cells in each group was determined with the use of 3-(4,5-dimethylthiazol-2-yl)-2, 5-diphenyltetrazolium bromide (MTT) assay. As illustrated in Figure 7, optical density (OD) values presented with insignificant statistical difference among groups at 1^st^ day (p > 0.05). Little significant difference was observed in cell viability between the blank group and the NC group at 1^st^, 2^nd^, 3^rd^, 4^th^, and 5^th^ days (p > 0.05). After 1 day, cell viability was increased in the miR-203 inhibitor group and reduced in the miR-203 mimic group and miR-203 mimic + XAV-939 group when compared with the blank and NC groups (p < 0.05). After 2 days, compared with the blank and NC groups, cell viability was decreased in the miR-203 mimic group and the XAV-939 group but elevated in the miR-203 inhibitor group (p < 0.05). However, no notable changes were detected in OD values among the blank, NC, miR-203 mimic + oe-PRC1, miR-203 inhibitor + sh-PRC1, and miR-203 inhibitor + XAV-939 groups (p > 0.05). Additionally, no significant difference of OD values was observed between the XAV-939 group and miR-203 mimic group (p > 0.05). After 2 days, cell viability was decreased in the miR-203 mimic + XAV-939 group as compared to the miR-203 mimic and XAV-939 groups (p < 0.05). Besides, the miR-203 mimic + oe-PRC1 group exhibited an enhancement of cell viability than the miR-203 mimic group, whereas the miR-203 inhibitor + sh-PRC1 group showed a reduction of cell viability as compared to the miR-203 inhibitor group (p < 0.05). These findings suggested that overexpressed miR-203 resulted in inhibited CSCC cell viability through downregulation of PRC1 and inhibition of the Wnt/β-catenin signaling pathway.

**Figure 7:** miR-203 Overexpression Inhibited the Proliferation of SCL-1 Cells ∗p < 0.05 versus the blank group and the NC group; #p < 0.05 versus the miR-203 mimic group and the XAV-939 group; and &p < 0.05 versus the miR-203 inhibitor group.

### Upregulated miR-203 Inhibits the Migration of SCL-1 Cells

Scratch test was used for the evaluation of migration potential of SCL-1 cells, the results of which (Figure 8) illustrated that with the prolongation of time, there was no statistical difference regarding cell migration in the NC, miR-203 mimic + oe-PRC1, miR-203 inhibitor + sh-PRC1, and miR-203 inhibitor + XAV-939 groups, relative to the blank group (p > 0.05). As compared to the blank group, cell migration was increased in the miR-203 inhibitor group and reduced in the miR-203 mimic and XAV-939 groups (p < 0.05). However, there was no significant difference found between the miR-203 mimic group and the XAV-939 group (p > 0.05). In comparison with the miR-203 mimic and XAV-939 miR-203 groups, cell migration in the miR-203 mimic + XAV-939 group was lowered (p < 0.05). Additionally, the miR-203 mimic + oe-PRC1 group exhibited an enhancement of cell migration than the miR-203 mimic group, whereas the miR-203 inhibitor + sh-PRC1 group showed a reduction of cell migration as compared to the miR-203 inhibitor group (p < 0.05). The aforementioned results indicated that the overexpression of miR-203 can repress the migration of the CSCC cells through downregulation of PRC1 and inhibition of the Wnt/β-catenin signaling pathway.

**Figure 8:** miR-203 Overexpression Inhibited the Migration of SCL-1 Cells (A) Representative images of SCL-1 cell migration distance measured using Scratch test. (B) Quantitative analysis of the number of migrated cells. ∗p < 0.05 versus the blank group and the NC group. #p < 0.05 versus the miR-203 mimic group and the XAV-939 group; and &p < 0.05 versus the miR-203 inhibitor group.

### Upregulated miR-203 Suppresses the Invasion of SCL-1 Cells

The invasion of SCL-1 cells was measured by Transwell assay. As illustrated in Figure 9, compared with the blank group, there was no significant difference in the NC, miR-203 mimic + oe-PRC1, miR-203 inhibitor + sh-PRC1, and miR-203 inhibitor + XAV-939 groups (p > 0.05). In comparison to the blank group, there was a significant elevation in cell invasion in the miR-203 inhibitor group and decrease in the miR-203 mimic and XAV-939 groups (p < 0.05). However, no difference was observed between the miR-203 mimic group and the XAV-939 group (p > 0.05). The invasive ability of cells in the miR-203 mimic + XAV-939 group was reduced when compared with that in the miR-203 mimic and XAV-939 groups (p < 0.05). Furthermore, the miR-203 mimic + oe-PRC1 group exhibited an enhancement of cell invasion than the miR-203 mimic group, whereas the miR-203 inhibitor + sh-PRC1 group showed an inhibition of cell invasion as compared to the miR-203 inhibitor group (p < 0.05). Thus, miR-203 was able to suppress invasion of the CSCC cells by targeting PRC1 and blocking the Wnt/β-catenin signaling pathway.

**Figure 9:** miR-203 Overexpression Restrained the Invasion of SCL-1 Cells (A) Representative images of cell invaded through the Matrigel (scale bar, 25 μm). (B) Quantitative analysis of the number of invasive cells measured by Transwell assay. ∗p < 0.05 versus the blank group and the NC group; #p < 0.05 versus the miR-203 mimic group and the XAV-939 group; and &p < 0.05 versus the miR-203 inhibitor group.

### Upregulated miR-203 Stimulates Apoptosis of SCL-1 Cells

The results from Annexin V/propidium iodide (PI) double staining (Figure 10) revealed that the apoptosis rates in the blank, NC, miR-203 inhibitor, miR-203 mimic, XAV-939, miR-203 mimic + XAV-939, miR-203 inhibitor + XAV-939, miR-203 mimic + oe-PRC1, and miR-203 inhibitor + sh-PRC1 groups at 48 h after transfection were 9.83% ± 0.91%, 9.71% ± 0.94%, 5.52% ± 0.47%, 17.54% ± 1.16%, 18.81% ± 1.21%, 32.31% ± 2.91%, 9.90% ± 0.87%, 9.85% ± 0.89%, and 9.82% ± 0.90%, respectively. Compared with the blank group, the apoptosis rate was lower in the miR-138 inhibitor group but higher in the miR-203 mimic group, the XAV-939 group and the miR-203 mimic + XAV-939 group (p < 0.05). Cell apoptosis was increased in the miR-203 mimic + XAV-939 group compared with the miR-203 mimic and XAV-939 groups (p < 0.05). In contrast to the miR-203 mimic group, the apoptosis rate was reduced in the miR-203 mimic + oe-PRC1 group (p < 0.05). However, the apoptosis rate was elevated in the miR-203 inhibitor + sh-PRC1 group relative to the miR-203 inhibitor group (p < 0.05). There was no significant difference in the rate of apoptosis observed among the blank, NC, miR-203 mimic + oe-PRC1, and miR-203 inhibitor + sh-PRC1, and miR-203 inhibitor + XAV-939 groups, as well as between miR-203 mimic group and the XAV-939 group (p > 0.05). In conclusion, overexpression of miR-203 promoted apoptosis of CSCC cells by targeting PRC1 and blocking the Wnt/β-catenin signaling pathway.

**Figure 10:** miR-203 Overexpression Promoted the Apoptosis of SCL-1 Cells (A) Flow cytometry scatterplot showing cell apoptosis. (B) Quantitative analysis of apoptosis rate. ∗p < 0.05 versus the blank group and the NC group; #p < 0.05 versus the miR-203 mimic group and the XAV-939 group; and &p < 0.05 versus the miR-203 inhibitor group.

## Discussion

CSCC is a major cause of cancer-related mortality in solid organ transplant recipients.^10^^,^^21^ miR-203 has been reported to act as a tumor-suppressive miRNA in numerous cancer types by targeting multiple coding genes.^10^^,^^22^ In this study, we found that upregulated miR-203 could potentially repress proliferation, invasion, migration, and promote apoptosis of CSCC cell line SCL-1 by blocking the Wnt/β-catenin signaling pathway via PRC1 downregulation.

Initially, our results showed a decrease in the expression of miR-203 and an increase in PRC1 expression in moderately and poorly differentiated CSCC tissues as compared to adjacent normal tissues, indicating that both miR-203 and PRC1 play significant roles in the initiation and progression of CSCC. A previous study screened out differentially expressed miRNAs in CSCC at different stages, the results of which showed that miR-203 tended to exhibit an upregulated expression pattern in well-differentiated CSCC, which was consisted with present findings.^9^ As reported by Lohcharoenkal et al.,^10^ miR-203 is downregulated in poorly differentiated tumor and restoring the low levels of miR-203 expression might provide therapeutic benefits, particularly in poorly differentiated CSCC. miR-203 is abundantly expressed in the skin and has been highlighted to have tumor-suppressive functions in other types of skin cancer, such as basal cell carcinoma.^23^^,^^24^. PRC1 has been reported to be aberrantly activated in human cancers such as breast cancer,^25^ hepatocellular carcinoma,^26^ and gastric carcinoma.^27^ Our study emphasized the key consideration that miR-203 and PRC1 are tightly associated with progression of CSCC.

Based on the results obtained from the target prediction online and luciferase activity, PRC1 was found to be a target of miR-203 and negatively regulated by miR-203. In our results, upregulated levels of miR-203 were accompanied by downregulated PRC1 expression. The ability of PRC1 to promote the assembly of microtubulin could potentially facilitate an increase in the stability of the spindle.^28^^,^^29^ Deregulation of PRC1 results in cytokinesis defects that facilitates chromosomal instability thereby contributing to tumor heterogeneity and cancer evolution.^30^ PRC1 exerts a promotive role in tumor progression in OSCC^31^ and gastric cancer.^27^ In addition, augmented expression of miR-203 leads to the inhibition of cell proliferation, migration, endothelial cell tube formation, and cancer stemness in prostate cancer through the suppression of its target gene SNAI2 (also known as Snail2).^32^ Also, Snail2 has been identified as a target of miR-203 in neural crest and hepatocellular carcinoma underlying the regulatory role of miR-203 in a wide range of biological processes.^33^^,^^34^ However, no difference was witnessed in Snail2 expression among moderately-, poorly-, and well-differentiated CSCC tissues and adjacent normal tissues. This disparity might be attributable to tumor heterogeneity. Here, we hypothesized that miR-203 exerted its tumor-suppressive role by targeting PRC1. We also found that the Wnt/β-catenin signaling pathway was activated in the presence of miR-203. The present study showed that the expression and distribution of PRC1 were dynamically regulated by the Wnt signaling pathway. PRC1 controlled the expression and function of WRRAGs like FANCI, SPC25, and KIF23 through the Wnt signaling pathway.^19^^,^^26^ Therefore, miR-203 might play a role as a cancer suppressor in CSCC cell line SCL-1 by targeting PRC1 and blocking the Wnt signaling pathway.

Subsequent assays revealed that the overexpression of miR-203 facilitated the apoptosis of CSCC cell line SCL-1, while suppressing proliferation, migration, and invasion by targeting PRC1 and blocking the Wnt/β-catenin signaling pathway. A previous study revealed that recovery of miR-203 induces cisplatin-induced tongue squamous cancer cell apoptosis and inhibits cell proliferation.^35^ There also may be a link between the aberrant activation of the Wnt/β-catenin signaling pathway and the development and progression of OSCC, as depicted in a pre-existing study.^15^ Hence, the Wnt/β-catenin signaling pathway might be a good target for cancer suppression. Yokogi et al.^36^ suggested that Wnt/β-catenin signal inhibitors might have the ability to decrease the number of OSCC stem cells and stimulate the tumor suppressive effect on OSCC cells. In agreement with our findings, miR-203 has been highlighted to attenuate the Wnt/β-catenin signaling pathway by targeting β-catenin, resulting in the inhibition of proliferation and migration of cancer stem cells.^37^ In addition, Chen et al.^26^ revealed that PRC1 expression, which adjusted the membrane isolation of the failure complex and stabilized the β-catenin by enhancing the degradation of APC, could be promoted by Wnt signaling pathway. Collectively, the above results suggested that PRC1 regulated the Wnt/β-catenin signaling pathway, which was controlled by miR-203. However, the function and underlying mechanism of action of PRC1 required further investigations.

In conclusion, on the basis of findings from our study that verified miR-203 as an anti-tumor miRNA in CSCC cell line SCL-1, we demonstrated that overexpression of miR-203 significantly promotes cell apoptosis and attenuates proliferation, migration, and invasion of CSCC cell line SCL-1 by targeting PRC1 and blocking the activation of Wnt/β-catenin signaling pathway (Figure S1). The aforementioned findings could potentially be used in the development of new therapeutic options for CSCC.

## Materials and Methods

### Ethics Statement

The study was conducted with the approval of the ethics committee of Peking Union Medical College Hospital. Informed written documents were obtained from all participants or their guardians prior to the study.

### Microarray-Based Gene-Expression Profiling

Data of GEO: GSE66359 dataset were retrieved in GEO database (https://www.ncbi.nlm.nih.gov/geo/) in National Center for Biotechnology Information (NCBI), a public platform for storing gene-expression datasets, original sequences, and records. It was found that GEO: GSE66359 included 8 cases of CSCC and 5 normal samples. The empirical Bayes method was used in the selection of the important differentially expressed genes in the Bioconductor based Limma package of R language. Finally, the differentially expressed genes were annotated by the Annotate package. p < 0.05 was considered statistically significant. The miRNA target prediction tools (miRSearch: https://www.exiqon.com/miRSearch, microRNA.org, http://www.mirdb.org/, and miRDB: http://mirdb.org/miRDB/index.html) were used to predict the miRNA that regulated candidate gene PRC1 and the intersection of the results was obtained. The expression of the PRC1 gene in the prognosis of CSCC was analyzed in The Cancer Genome Atlas (TCGA) database (http://ualcan.path.uab.edu/cgi-bin/ualcan-res.pl).

### Study Subjects

The cancer tissues and normal adjacent tissues were collected from 36 patients who had received a definite CSCC diagnosis at the dermatological department of Peking Union Medical College Hospital from November 2014 to April 2016. Tissue samples were then stored at −80°C. The patients consisted of 25 males and 11 females aged 40–76 years with the mean age of 55.4 years. The CSCC patients included in this study were categorized using the classification standard proposed by Albert Compton Broders,^38^ among which 10 were stage I were with highly differentiated CSCC, 19 were stage II with moderately differentiated CSCC, and 7 were stage III–IV with poorly differentiated CSCC. The inclusion criteria were as follows: patients were diagnosed with CSCC by tumor pathology and genetics and patients had resectable tumor based on clinical evaluation. None of the included patients received any chemotherapy, radiotherapy, or other anti-tumor treatments before the operation. The patients were excluded when diagnosed with CSCC before November 2014, with other cancers or with autoimmune disease, immunosuppressive disease, or other skin diseases (psoriasis).

### Dual-Luciferase Reporter Gene Assay

microRNA.org prediction website was used for the analysis of the target gene of miR-203. The bioinformatics was applied to predict the target binding site of miR-203 and PRC1 gene. Synthesized primers were obtained from Shanghai GeneChem (Shanghai, China). The WT vector was constructed as follows: amplified 3′ UTR sequence of PRC1 was cloned and inserted in pmiR-RB-REPORT vector digested by restrictive endonuclease XhoI/NotI. The MUT vector was constructed with WT vector used as a template. MUT primers were designed and two mutation subsections were obtained by PCR, and lastly the products of PCR were purified and cleaved by restrictive endonucleases XhoI/NotI, which were harvested and inserted into pmiR-RB-REPORT vector. The generated PRC1-MT or PRC1-MUT plasmid was co-transfected with miR-203 mimic into SCL-1 cells (Guangzhou Jennio Biotech, Guangdong, China), followed by luciferase activity detection at 560 nm with the use of a Firefly Luciferase Reporter Gene Assay Kit (RG005, Beyotime Biotechnology, Shanghai, China) and a microplate reader (MK3, Thermo Fisher Scientific, Waltham, MA, USA). The miScript target protectors were modified RNA oligonucleotides complementary to specific target sites that could not bind to other sequences.^39^

### Immunohistochemistry

Human CSCC tissues and adjacent normal tissues were fixed in 4% paraformaldehyde and decalcified with 10% ethylenediaminetetraacetic acid (EDTA). The tissues were conventionally dehydrated, cleared, immersed by wax, embedded into paraffin, and cut into 4-μm-thick sections. The sections were then conventionally dewaxed by xylene I and II, respectively, each for 10 min, and dehydrated with gradient alcohol of 100%, 95%, and 85%, each for 2 min. Following antigen retrieval at high temperature for 90 s, the sections were cooled down, and incubation was carried out with 3% H_2_O_2_ for 5–10 min for the removal of endogenous peroxidase activity. Then the sections were added with 50 μL of non-immune animal serum and placed in a wet box for 5 min of incubation. The sections were added with rabbit anti-human monoclonal antibody to PRC1 (1: 200, ab51248, Abcam, Cambridge, UK) at 4°C for 12 h, followed by the addition of biotin-labeled secondary antibody for incubation for 30 min. Then the sections were added with streptavidin-peroxidase for 10 min and added with freshly prepared diaminobenzidine (DAB) mixed dye liquor for 10 min of staining with the avoidance of light exposure. Development was carried out under a microscope. After full development, the sections were washed under running water, counter-stained by hematoxylin for 5 min, washed again under running water for 10 min, dehydrated with gradient alcohol, cleared with xylene, mounted with neutral balsam, and covered with coverslips. The tissues presenting blue or light blue were regarded as negative and those with brownish yellow granules were positive. Three non-overlapping visual fields were randomly selected, and the Nikon Image analysis software (Nikon Vision, Tokyo, Japan) was used to calculate the number of positive cells for each slice, using the following formula: percentage of positive cells = number of positive cells/total cell number × 100%.

### *In Situ* Hybridization

*In situ* hybridization was carried out to determine the transcriptional level of miR-203 in the frozen skin tissue sections collected from patients with invasive CSCC. Briefly, the sections were hybridized with miRCURY LNA probes (Exiqon, Woburn, MA, USA) labeled with digoxygenin overnight, followed by incubation with alkaline phosphatase-conjugated antibody to digoxygenin at 4°C overnight. Alkaline phosphatase reaction was performed in polyvinyl alcohol (PVA) with MgCl_2_ and NBT/BCIP (Roche, Florence, SC, USA). Digoxygenin-labeled-locked nucleic acid miR scramble (Exiqon, Woburn, MA, USA) was used as controls for hybridization. Images were subsequently captured using Nikon Eclipse E400Q imaging camera (Nikon, Tokyo, Japan) and analyzed with the use of NIS-Elements’ BR 3.10 software.

### Cell Culture, Grouping, and Transfection

Human CSCC cell line SCL-1 (Guangzhou Jennio Biotech, Guangzhou, China) was cultured in Dulbecco’s modified Eagle’s medium (DMEM; GIBCO Biotech, CA, USA) containing 10% fetal bovine serum (FBS). The cells were seeded in a 6-well plate at a density of 2.5 × 10^5^ cells/well and cultured with 5% CO_2_ at 37°C. Following attachment, the cells were treated with 0.25% trypsin and passaged. Cells at the phase of logarithmic growth were selected for subsequent experiments. The sequences of NC, miR-203 mimic, and miR-203 inhibitor (Table 1) were synthesized by Switch Gear Genomics (Menlo Park, CA, USA). The mature miR-203 sequence driven by CMV promoter and EmGFP reporter gene driven by CMV promoter were inserted into pGCMV/EGFP/miR/Blasticidin vectors to generate miR-203 mimic and miR-203 inhibitor, respectively. Subsequently, the cells were classified into the blank group (no plasmid transfection), NC group (cells transfected with NC plasmid), miR-203 mimic group (cells transfected with miR-203 mimic), miR-203 inhibitor group (cells transfected with miR-203 inhibitor), XAV-939 group (cells treated with XAV-939, an inhibitor of the Wnt/β-catenin signaling pathway), miR-203 inhibitor + sh-PRC1 group (cells co-transfected with miR-203 inhibitor and shRNA targeting PRC1), miR-203 mimic + oe-PRC1 group (cells co-transfected with miR-203 mimic and oe-PRC1), miR-203 mimic + XAV-939 group (cells transfected with miR-203 mimic and treated with XAV-939), and miR-203 inhibitor + XAV-939 group (cells transfected with miR-203 inhibitor and treated with XAV-939). Tankyrase inhibitor, XAV-939 (MedChemExpress, NJ, USA), has been reported to induce Axin stabilization and to cause subsequent destruction of the β-catenin complex and dephosphorylation of β-catenin.^40^ Prior to transfection, cells at the logarithmic growth phase were seeded in a 6-well plate. When density reached 80%–90%, the cells underwent centrifugation at 179 × *g* for 5 min and were transferred into serum-free Roswell Park Memorial Institute (RPMI) 1640 medium for culture. Afterward, the cells were transfected using Lipofectamine 2000 transfection reagent. Each 6-well plate was added with 500 μL solution C, mixed evenly, and cultured together with 5% CO_2_ at 37°C. After 6 h, the original medium was replaced by complete RPMI 1640 medium and cultured for additional 24 h. Then the G418 (Amersco Biotech, Solon, OH, USA) with the density of 400 μg/mL was used to screen cells. After 2–3 weeks, when monoclonal cells can be clearly distinguished with the naked eyes, the monoclonal clones were amplified and cultured in the RPMI 1640 medium to establish a stably transfected monoclonal cell line.

**Table 1:** Primer Sequences of Negative Control Plasmid, miR-203 Mimic, and miR-203 Inhibitor

Plasmid	Primer Sequence
Negative control plasmid	5′-UCACAACCUCCUAGAAAGAGUAGA-3′
miR-203 mimic	5′-GUGAAAUGUUUAGGACCACUAG-3′
miR-203 inhibitor	5′-GUGAAAUGUUUAGGACCACUAG-3′

miR-203, microRNA-203.

### RNA Isolation and qRT-PCR

Total RNA was extracted from cells transfected for 24 h with TRIzol (Invitrogen, Carlsbad, CA, USA). Spectrophotometry and agarose gel electrophoresis were used to evaluate the concentration, purity, and integrity of the extracted RNA. The primers were synthesized by Shanghai Sangon Biotech (Shanghai, China; Table 2). For miRNA expression determination, one μL RNA was reversely transcribed by using miScript Reverse Transcription Kit (QIAGEN Company, Duesseldorf, Germany), and subjected to quantitative real time PCR using SYBR Green PCR Master Mix (Takara Holdings, Kyoto, Japan) with U6 serving as internal reference. The reaction system consisted of 10 μL SYBR Green Master Mix, 0.5 μL miR-specific stem-loop primers (Applied Biosystems, Carlsbad, CA, USA), 0.5 μL universal adaptor PCR Primer, 2 μL DNA template, and 7 μL ddH_2_O. For gene expression determination, complementary DNA (cDNA) was generated using a qScript cDNA Synthesis kit (Quanta BioSciences, Gaithersburg, MD, USA) and quantitative real time PCR was run in triplicates using the PerfeCTa SYBR Green SuperMix (Quanta BioSciences, Gaithersburg, MD, USA) with β-actin used as a reference gene.^41^ 2^-ΔCT^ method was used for qRT-PCR data analysis.

**Table 2:** The Primer Sequences of miR-203, U6, PRC1, β-actin, β-catenin, Wnt8b, c-Jun, FZD3, p16, Bcl-2, and c-Myc used for qRT-PCR

Gene	Sequence
miR-203	F: 5′-TGCTCTAGAGGCGTCTAAGGCGTCCG-3′
	R: 5′-CCCAAGCTTCACCTCCCAGCAGCACTTG-3′
U6	F: 5′-AAAGCAAATCATCGGACGACC-3′
	R: 5′-GTACAACACATTGTTTCCTCGGA-3′
PRC1	F: 5′-CAAGCGCCGTATGGGACTTT-3′
	R: 5′-GGAGGCATCCATGTAGCTCT-3′
β-actin	F: 5′-AGCGAGCATCCCCCAAAGTT-3′
	R: 5′-GGGCACGAAGGCTCATCATT-3′
β-catenin	F: 5′-GCAACCCTGAGGAAGAAGAT-3′
	R: 5′-TTAGCTCCTTCCTGATGGAG-3′
Wnt8b	F: 5′-CCGACACCTTTCGCTCCATC-3′
	R: 5′-CAGCCCTAGCGTTTTGTTCTC-3′
c-Jun	F: 5′-AAAGAATTCATGACTGCAAAGATGGAAACG-3′
	R: 5′-AAACTCGAGTCAAAATGTTTGCAACTGCTG-3′
FZD3	F: 5′-GTTCATGGGGCATATAGGTGG-3′
	R: 5′-GCTGCTGTCTGTTGGTCATAA-3′
p16	F: 5′-TGTGTCCAGTCCATGCCAAC-3′
	R: 5′-AGGAAATCGTAGCACTGCAAG-3′
Bcl-2	F: 5′-GTCTTCGCTGCGGAGATCAT-3′
	R: 5′-CATTCCGATATACGCTGGGAC-3′
c-Myc	F: 5′-ATGGCCCATTACAAAGCCG-3′
	R: 5′-TTTCTGGAGTAGCAGCTCCTAA-3′
Snail	F: 5′-TCCAGAGTTTACCTTCCAGCA-3′
	R: 5′-CTTTCCCACTGTCCTCATCTG-3′

qRT-PCR, quantitative reverse transcription polymerase chain reaction; miR-203, microRNA-203; PRC1, polycomb repressive complex 1; FZD3, frizzled-3; Bcl-2, B cell leukemia/lymphoma 2; F, forward; R, reverse.

### Western Blot Analysis

After 48 h of transfection, the cells were collected, washed twice with PBS following medium removal, placed on ice, and fully cracked by radioimmunoprecipitation assay lysis buffer (P0013B, Beyotime Biotechnology, Shanghai, China) supplemented with protease inhibitor. The protein concentration was determined with bicinchoninic acid (BCA). The protein was then separated by sodium dodecyl sulfate polyacrylamide gel electrophoresis (SDS-PAGE) and transferred onto polyvinylidene fluoride (PVDF) membranes by a semi-dry membrane apparatus and blocked for 2 h with phosphate buffered saline Tween-20 (PBST) containing 5% skimmed milk powder. The membrane underwent incubation overnight at 4°C with the following primary antibodies diluted at ratio of 1:1,000 and purchased from Abcam, Cambridge, MA, USA: rabbit anti-human PRC1 (ab140033), β-actin (ab8226), β-catenin (ab16051), Wnt8b (ab66307), c-Jun (ab31367), FZD3 (ab75233), p16 (ab151303), Bcl-2 (ab32124), and c-*myc* (ab32072). The membrane was then washed 3 times (15 min each time) by 20 mM Tris-HCl, 150 mM NaCl, and 20mM 0.05% Tween 20 (TBST) solution and incubated with secondary antibody horseradish peroxidase (HRP)-labeled goat anti-rabbit immunoglobulin G (IgG; 1:1,000, Santa Cruz Biotechnology, Santa Cruz, CA, USA). Following a 2 h incubation at room temperature, the membrane was washed with the TBST 3 times (each time for 15 min), followed by visualization with enhanced chemiluminescence (ECL) reagent for 2 min. Band intensities were quantified using an Image-Pro Plus 6.0 software. The relative protein expression was regarded as the ratio of the gray value of the target band to β-actin.

### MTT Assay

The cells were rinsed twice by PBS after SCL-1 cell density reached approximately 80% and received treatment with 0.25% trypsin to form single cell suspension. After counting, the cells were shifted to a 96-well plate with 5 × 10^3^ cells/well (5 replicates were ready), and the volume of each well was 200 μL. After culture for 48 h, each well was added with 20 μL MTT liquid (5 mg/mL, A2776-1G, Shanghai Shi Feng Biotechnology, Shanghai, China) and cultured for 4 h. After the culture solution in the wells was suctioned out with the use of a 5 mL injector, 150 μL DMSO was added into each well for low-speed oscillation on a shaker for 10 min. OD value was measured in each well at 490 nm using a microplate reader when the cells were cultured for 1–6 days. The growth curve was plotted with time as the x axis and OD as the y axis. The experiment was conducted in triplicates.

### Scratch Test

Cell counting was carried out after the SCL-1 cells at logarithmic growth phrase were treated with trypsin evenly and fully re-suspended. The cells were diluted to 1 × 10^5^ cells/well and seeded to 24-well culture plates followed by addition with medium containing 10% FBS, followed by culture in 5% CO_2_ at 37°C. After the cells grew into single layer, the medium was sucked away and a straight thin wound was created at the bottom of the 24-well plate at the center of the single cell with a 200 μL sterile pipette tip. The scratched cells were washed away with PBS, and the remaining cells were added with serum-free medium and cultured in 5% CO_2_ at 37°C. Images were obtained at the same position when cultured for 0 h, 24 h, and 48 h. Three replicated wells in each group were set for observing the “healing” of the wounds and the migration ratio was calculated as follows: migration ratio = (V_T0_ - V_Tt_) / V_T0_ × 100%.^42^

### Transwell Assay

The Matrigel was prepared by serum-free DMEM (medium: Matrigel = 3: 1), gently oscillated, and placed in the inner side of Transwell chamber (3413, Millipore, Billerica, MA, USA) at 37°C for 2 h. Before usage, the gel was hydrated by the addition with a small amount of serum-free medium. SCL-1 cells at the logarithmic growth phase were detached using trypsin, and centrifugation was carried out at 28 × *g* for 5 min at room temperature with supernatant discarded, followed by one wash and re-suspension in serum-free DMEM. A total of 1 × 10^6^ cells were seeded into Transwell apical chamber. The basolateral chamber was incubated with 500 μL DMEM containing 20% FBS with 3 replicates in each group for 48 h. The cells were fixed for 30 min with 4% paraformaldehyde after the removal of the Transwell chamber. The cells were rinsed by PBS and stained with Giemsa for 20 min. The Matrigel at the bottom of the apical chamber and the non-invasive cells were wiped out with cotton swabs. The Transwell chamber was inverted, observed, and photographed under an optical microscope. The invaded cells were counted in 10 randomly selected low and high visual fields. The experiment was conducted in triplicates. The number of cells passing through the Matrigel indicated the invasion ability of cells.

### Annexin V-Fluorescein Isothiocyanate (FITC)/PI Double Staining

After 48 h of transfection, the cells underwent incubation with 0.25% trypsin and centrifugation, followed by supernatant removal. The cells were added with 5 mL 70% ethanol solution, placed at 4°C for 48 h, and centrifuged (17,891 × *g* for 5 min) after being washed with PBS. After being washed with PBS, the cell clusters were broken down using 1 mL PBS, added with 5 μL hydrolase RNase (10 mg/mL), and allowed to stand at 37°C for 1 h. Then, 100 μL cell suspension was added with 5 μL Annexin V-FITC and 2.5 μL PI, mixed gently and uniformly and incubated for 30 min avoiding light exposure before examination using flow cytometer. The percentage of apoptotic cells was calculated using the CellQuest3.0 software.

### Statistical Analysis

Statistical analysis was conducted using SPSS 21.0 (IBM, Armonk, NY, USA). Measurement data were expressed as mean ± standard deviation. Comparison among multiple groups was conducted by one-way or two-way analysis of variance (ANOVA) and the variance homogeneity test was implemented. Comparison between two groups was conducted using the Q test if the data obeyed homogeneity of variance, and differences were compared by the nonparametric rank-sum test when homogeneity of variance was violated. With α = 0.05 as test standard, p <0.05 was regarded as statistically significant. The enumeration data were expressed as percentages or ratios, and X2 test was used for comparison.

## Author Contributions

W.T. and C.F. designed the study. M.Z. collated the data, carried out data analyses, and produced the initial draft of the manuscript. F.L. and M.B. contributed to drafting the manuscript. All authors read and approved the final manuscript.

## Conflicts of Interest

The authors declare no competing interests.

## Supplemental Information

Table S1. MicroRNA

Table S2. miRDB

Table S3. miRSearch
